The article "Interpretation of Online Artworks of Digital Art Design in the New Media Environment" was published in 2022. Journal: J Environ Public Health.

# Interpretation of Online Artworks of Digital Art Design in the New Media Environment

**DOI:** 10.1155/2022/9566844

**Published:** 2022-06-20

**Authors:** Pingping Li

**Affiliations:** Zhengzhou Normal University, Zhengzhou, Henan 450000, China

## Abstract

In order to realize the interpretation of online artworks, the art design of artworks is studied on the basis of new media digital environment. Through the presentation of digital works, the enhancement of dramatic art appreciation, the balanced display of art appreciation, and the enhancement of digital aesthetic creation, the interpretation of artworks has been successfully completed, which strongly supports the digitization of new media. Art design is to constantly breed an updated online art space and attract and summon more viewers' new experience, new creation, and new perception so as to trigger and develop new propositions, new exploration, and new atmosphere of new media drama. For the current construction of traditional art design, new media digital technology plays a major role. The transformation of digital technology and Internet media is another “holographic” extension of the human body, which has an extremely strong impact on new media art and comprehensively updated our life, art, and aesthetic concepts. This is not only a revolution of media but also a change of art. At the same time, it is also accompanied by the “expansion” of art theory. What this change ultimately needs to complete is the revolution of media culture that affects the development process of human civilization.

## 1. Introduction

The rapid development of digital technology has had a wide impact on the whole industrial chain, such as the production, dissemination, and acceptance of new media art. Particularly after entering the 21st century, the speed of high-tech renewal and iteration has accelerated, and new media art has undergone all-round changes, including the changes of aesthetic concepts and art theories. New media art, in a broad sense, is based on digital technology and digital image as the media, including films accepted by the art system as the “seventh art,” television as the “eighth art,” and games as the “ninth art,” as well as many art forms related to film and television art, such as 3D image, VR image, and video game fusion image. New media art provides us with a new aesthetic experience mode. New media have brought about fundamental changes in aesthetic experience and changed from the dominant mode of self-sufficient object perception to the mode with specific emotional intensity as the core. To some extent, new media make our internal movement, which proves once again their essential creativity. In the environment of “experience economy,” the online artworks of new media drama need “role breakthrough.” The stronger audience's drama experience is reflected in the strengthening of audience experience consciousness in traditional drama, the in-depth exploration of audience experience in cutting-edge drama, and the expansion of audience drama experience by new media performance. After the beginning of the “experience economy era,” the evolution of audience experience of new media drama has evolved from “strong interaction” to “strong recognition” and from “passive participation” to “active creation.” The drama experience space has appeared as “extension” and “regeneration,” and the connotation of drama experience has also appeared as “transformation” and “sublimation.” “Audience drama experience evolution” promotes the role breakthrough of new media drama online artworks. In the era of “experience economy,” new media drama online artworks have increased, enriched, and changed their roles. “Dance role breakthrough” directly leads to the innovation of experiential dance space in new media drama. “Audience's deep drama experience demand” is the basic driving force for the transformation of new media drama experiential dance space. “Dance role evolution” is not only the starting point but also the end point of promoting the innovation of experiential dance space in new media drama. “Unfinished space” is the soil that breeds new media drama experiential online art works.  Figure 1 is an analysis of digital self-media in the field. Equilibrium can be regarded as the basis of all aesthetic principles, and other principles can be regarded as the derivation of this basic principle.

The article "Interpretation of Online Artworks of Digital Art Design in the New Media Environment" was published in 2022. Journal: J Environ Public Health.

## 2. Literature Review

Yoo C. et al. said that the progress of digital technology not only provides a development opportunity for film and television media and film and television art but also has a strong impact on the whole “great art” theoretical system, including film and television art and other new media arts. To some extent, the process of art development is the process of continuous “expansion” of art theory [1]. Zhang G. et al. believe that “new media” has become a popular term in society, and “new media drama” has also become a hot topic in the drama circle. In the past two decades, the exploration and creation of new media drama in China have not brought a considerable scene for its prosperity. On the contrary, with the proliferation of forms or the increase of gimmicks to a certain extent, it has become controversial, and the voice of doubt and opposition seems to be even more [2]. Glava Z. et al. believe that many discussions on digital media art design focus on the application of technical tools while ignoring its artistic and cultural spirit. Therefore, we want to use the modern digital technology platform to integrate Chinese elements into digital media art design, which not only enriches the design elements but also can use the digital media communication platform to better show the brilliance of Chinese art and culture [3]. Wang X. et al. said that although digital art design has been widely used in various fields of our life because of its unique charm and nature, there is still a lack of complete theoretical system support for digital art design [4]. Therefore, Song M. et al. believe that online art works should first have the characteristics of disseminating information and visual stimulation. The so-called “visual stimulation” refers to the visual psychological process of attracting the audience's interest and naturally generating three steps in an instant, namely, stimulation, communication, and impression. “Stimulation” is to make the audience pay attention to it, “transmission” is to convey the information to the audience as soon as possible, and “impression” is the content expressed to form an image memory for the audience [5]. Bruhn J. et al. believe that, under the background of new media, the communication technology, communication carrier, and users' reading preference of news have changed to some extent. More and more elements participate in the process of art creation and communication. News writing presents different writing characteristics, and aesthetic art also permeates the process. Three-dimensional, visual, and storytelling are not only the aesthetic and artistic embodiment of new media online writing but also the transformation direction of art writing [6]. Therefore, while Gorbunova A. et al. have accumulated teaching experience, in the new media era, the coverage of news content is closely related to technology and information collection ability. Usually, in order to seize the opportunity, the news reports in the context of new media are simple and direct, but with the increasing attention of users and the mining of relevant news elements [7]. Y. Xu et al. said that the new aesthetics brought by the new media art based on digital technology and with digital image as the core has opened a new era of film and television art and image culture and put forward new challenges for the original art theory system and aesthetic system with classical art as the main interpretation object [8]. Wakelin Daniel Iyer G. et al. believe that, at this stage, there are obviously problems that need to explored, thought of, or solved. Based on the dual-era environment of “new media” and “experience economy,” they focus on the perspective of online artworks of new media drama [9]. Bellalouna F. et al. believe that, under the background of “globalization” of digital information, with the development of economy and the renewal of technology, digital technology is involved in the field of art, produces computer graphics and image design works, and then is involved in dynamic film and television and digital interactive design works. After digital technology enters the art field, the boundary between “pure art” and “commercial design” becomes more and more blurred [10].

The article "Interpretation of Online Artworks of Digital Art Design in the New Media Environment" was published in 2022. Journal: J Environ Public Health.

## 3. Method

### 3.1. Presentation of Digital Artworks

Digital media art design is a new means of expression of today's digital art design. In order to better show China's original culture and artistic characteristics under the background of international globalization, the selection and application of Chinese elements is the innovation and development of today's digital information media. Therefore, the use of digital media to show Chinese elements can better show and develop Chinese art and culture. Therefore, the perfect integration of Chinese art and digital technology can form a certain psychological formula and finally show the digital media art design with the style of Chinese national art and culture. This attempt not only shows the digital media art design with the Chinese national art design style but also provides some experimental exploration experience for the style creativity of more digital media art design in the future [11]. Reflecting the brand of Chinese national culture and making it occupy a place in the forest of world culture is an urgent problem to be considered in modern digital media art design because only the national is the world. The elements of digital media art design should reflect Chinese traditional culture and constantly improve the quality and cultivation of designers. Based on the platform provided by new technology, we use the modern digital expression to integrate traditional Chinese elements into digital. Without the intervention of external forces, it will develop self-sufficient and healthy so as to approach the essence of art infinitely.  Figure 2 is the flowchart of the new media operation, and Figure 3 is the composition of the new media digital team. However, too much use of ideological standards to measure artistic creation and aesthetic thought has brought artificial class nature to aesthetics and art. At the same time, during this period, academic research was stagnant, resulting in many thinking achievements of intellectuals being “dead in the womb” and failed to appear. Based on this lesson, in the new era, we should put the discussion of art and aesthetic theory back to the field of academic research, talk about academic research, and provide “green” protection for the healthy development of academics so as to promote the emergence and birth of important aesthetic and artistic theory works in the new era [12].

The article "Interpretation of Online Artworks of Digital Art Design in the New Media Environment" was published in 2022. Journal: J Environ Public Health.

In addition to the big movies watched on the big screen, as far as other new media arts in different forms are concerned, digital images have penetrated into all aspects of our daily life, and the digital images transmitted on all kinds of new media together constitute our daily life. This makes aesthetic elements integrated into daily life, and daily life can also be easily transformed into image content, which has achieved “aestheticization of daily life.” New media art image has become “a fast stream of symbols and images filled with the longitude and latitude of daily life in contemporary society” [13].  Figure 4 shows the overall market scale of new media server. In this kind of image consumption behavior, the boundary between elegant art and popular art has been erased, the classical aesthetic order and artistic level have been disintegrated, the sense of sanctity of art appreciation no longer exists, and the traditional aesthetic attitude of watching quietly has gradually disappeared as the “sense of distance” between daily life and the traditional sense of film viewing ceremony. As shown in Figure 5, the propagation speed formula (1) of new media under digitization is as follows:

(1) $$\begin{array}{c} v=\frac{n}{d}, \end{array}$$

where *d* represents the communication duration, *n* represents the total number of news within the communication duration, and *v* represents the communication speed. The communication duration, communication speed, and target group coverage need to be normalized. Taking the propagation time as the target, the formula is

(2) $$\begin{array}{c} T=\frac{1}{1+e^{-t}}. \end{array}$$

According to the digital media, we can get the output formula of the design terminal under the new media environment as follows:

(3) $$\begin{array}{c} E=\frac{1}{2}{\left(d-o\right)}^{2}. \end{array}$$

### 3.2. Enhance the Appreciation of Dramatic Art

“The evolution of dance role” is not only the starting point but also the end point of promoting the innovation of experiential dance space in new media drama. In the new media drama, the role of stage art gradually presents multipolarization, that is, “behind the scenes” role, “script” role, “character” and “actor” role, and “director” role. Besides the “behind the scenes” role, other roles are becoming more and more important, and some roles even play a decisive role in the benign development of new media drama [14], for example, the role of “actor” and “director”; the extension or transformation of the stage art role of this kind of drama is almost difficult to see in the past traditional drama performance, which is unimaginable for the current formal or routine new media drama, and may also be based on the “actor-centered theory.” “Director-centered theory” for the singing tone of the dramatic art actor or director is unwilling to imagine. In any case, the continuous embarrassment and confusion of new media drama are prompting us to think about “change,” “change when poor, change when flexible, and general for a long time.” The proposition of stage art of new media drama is changing, and the action of breaking the topic is bound to change. If we still use the old method to solve the new proposition, we can imagine its future. The evolution of the role of dance beauty just promotes the effective formation of the experiential dance beauty space of new media drama, forces the drama and dance beauty to move further towards the direction of audience space experience, provides a richer and more favorable platform for audience drama experience, and contains unlimited opportunities for “integrating drama space.” It is in this experiential dance beauty space that the audience obtains a new understanding, then promotes the “evolution of dance beauty roles” at a higher and broader level, and continuously promotes the experiential dance beauty space into a higher level of space. It goes without saying that “dance role evolution” is not only the starting point of promoting the innovation of new media drama experiential dance space but also the end point of innovation and always makes an unlimited expedition to a higher level of “starting point” and “end point,” which will be the necessary way for the return of the noumenon of “inclusive drama space” [15].  Figure 6 shows the crisis management module for digital art interpretation.

The article "Interpretation of Online Artworks of Digital Art Design in the New Media Environment" was published in 2022. Journal: J Environ Public Health.

The crisis management module is the main module of the system, which mainly realizes a series of processes in the place of digital art interpretation to ensure the value of artworks. The realization of this function directly affects the overall effect of works [16]. The flowchart of online art appreciation is shown in Figure 7.

Better integrate Chinese art and digital technology to form a certain psychological formula, and finally show the digital media art design with Chinese national art and cultural style. This attempt not only shows the digital media art design with the Chinese national art design style but also provides some experimental exploration experience for the style creativity of more digital media art design in the future. Reflecting the brand of Chinese national culture and making it occupy a place in the forest of world culture is an urgent problem to be considered in the art design of modern digital media [17]. The problems of modern digital media art design are shown in Figure 8.

The test and evaluation module is mainly used to test the interpretation of online artworks. It is an intuitive evaluation of digital new media. The main function of this module is phased inspection: phased inspection is to ensure the correct online interpretation of artworks [18]. The test evaluation module is shown in Figure 9.

User communication module is an important functional module to realize the interaction between new media management and art communication personnel in the process of art teaching activities. It is mainly used for information exchange activities between users. The module mainly includes real-time interactive online Q & A and online messages. Before answering questions, the work personnel need to create a Q & A room, and the enterprise personnel can answer questions in real time after entering the corresponding Q & A room so that they can answer questions in groups in different places and classes at the same time [19]. The user communication module is shown in Figure 10.

The system management module mainly manages user accounts, including adding users, deleting users, and modifying user information, and can assign permissions to users at the same time. System parameters can be maintained, and system data can be backed up. The function module of the background management module is shown in Figure 11.

### 3.3. Balanced Display of Art Appreciation

The reason why balance is called the most basic aesthetic principle is that it originates from the original heart and conforms to our most simple and classical aesthetic norms. It can best comfort the viewer's psychology and make the viewer feel comfortable and safe, just as we often say: “stability is the foundation of everything.” With symmetry and balance, there is the foundation of beauty. Other aesthetic principles are the variation and derivation on this basis. Balance is to make the picture feel a physical balance psychologically through our eyes through the placement and combination of various elements. Balance is different from symmetry. Symmetry gives people the feeling of “preciseness and solemnity” through formal equality, similarity, and similarity, while balance makes the picture feel “stable” through appropriate combination [20]. Balance: there are two forms: symmetric balance and asymmetric balance. Symmetrical balance is called “axisymmetric” balance. “Axis” refers to the equal weight on both sides, giving people a sense of security, stability, and solemnity. Asymmetric equilibrium means that the components on both sides of the “axis” are not equal. Using the visual law, the components on both sides of the “axis” are adjusted by changing the size, shape, distance, density, and other factors, giving people a sense of balance. This form gives people a feeling of novelty, liveliness, and strong sense of movement and has a certain appeal [21].  Figure 12 shows the balance principle of online artworks.

The article "Interpretation of Online Artworks of Digital Art Design in the New Media Environment" was published in 2022. Journal: J Environ Public Health.

### 3.4. Enhance Digital Aesthetic Creation

The creation of art design is a process of image conception and materialization. This process requires the creator's spiritual feelings and the accumulation of creative experience to form his own thinking. Specifically, this includes two aspects: first, the creation of art design is a process in which the creator constructs images through spiritual feelings. The “image” here not only has an aesthetic function but also permeates the specific content of social culture and contains a variety of ideas, such as politics and religion, emotion and action, mood, and expression. From this perspective, the creation of art design is the unity of image and concept [22].  Figure 13 shows the number of recent online artworks. Secondly, the creation of art design also needs the creator's personal ability and computer skills because the materialization process of “image” must be realized through design skills, such as shape, color, and texture, which is an indispensable process of forming realistic art design works. From the above description, we can know that the creation mode of art design is related to the type of design object and the personality of the creator, so there is no common model. However, the creation of art design should also follow certain laws and conform to the universality of contradictions [23].  Figure 14 shows the artistic image of online artworks. Because different artistic design creation processes must go deep into life, collect images in personal ideas so as to stimulate the creator's creative desire and materialize the “image” in time, which is the communication process of artistic design. After computers are widely used and mankind has entered the digital era, the great influence of computers on the creative methods of art design has further deepened the creation on the original basis and formed creative methods with their own characteristics, such as algorithmic creation, simulation creation, combination of algorithmic and imitation creation, virtual reality creation, and automatic creation. The error matrix sent by the new media according to the system is shown in formula (4):

(4) $$\begin{array}{c} \overset{2}{\underset{f}{\left(Y-DX\right)}}=\overset{2}{\underset{f}{\left(E_{K}-d_{k}\overset{k}{\underset{r}{x}}\right)}}. \end{array}$$

Among them, we only need to adjust *d*_*k*_ and *x*_*r*_^*k*^ to realize the minimum solution of error.

The article "Interpretation of Online Artworks of Digital Art Design in the New Media Environment" was published in 2022. Journal: J Environ Public Health.

### 3.5. Realize New Media Art Interpretation

New media drama experience also includes the drama experience of the audience. This kind of experience seems to be difficult to see in the existing new media drama exploration or works. More often, it is the feeling of self-entertainment of new media, which is still a long way from the truly integrated drama. To a large extent, the audience's drama experience needs to be based on the online artworks of new media drama. Without its online artworks, the audience's drama experience and inclusive drama can hardly be realized.  Figure 15 shows the audience satisfaction survey of new media art interpretation. Therefore, in order to realize the effective development of new media drama, the drama experience space of its online artworks is the cornerstone and focus [24]. If new media drama leaves the drama experience space of online artworks, ignores the drama experience role of online artworks, or does not tap the rich drama experience of online artworks, it will be difficult to achieve the vigorous development of new media drama. The experiential stage art of new media drama is an indispensable link in the benign development of new media drama. As shown in Figure 16, the reading volume of dramatic artworks is compared with that of previous works. In media art design, the digital media art design is endowed with cultural connotation, and digital expression is used to reproduce the brilliance of China's traditional art.

At the same time, the digital media art design is a new means of expression of today's digital art design. In order to better show the original cultural and artistic characteristics under the background of international globalization, the selection and application of Chinese elements is the innovation and development of today's digital information media. Therefore, using digital media to show Chinese elements can better show and reduce the difference between Chinese art and culture. Only with the support of a complete theoretical system can we produce scientific ideas and concepts of digital art design. Under the guidance of these thoughts and thoughts, we can really go deep into the creation and appreciation of digital art and design so as to break through the shackles of traditional mode and give full play to the charm of digital art and design [25]. Viewing digital art and design from the fields related to our vision, we can find that digital art and design has penetrated into our lives, from electronic products to colorful web pages on the Internet and from a large number of stunts used in commercial blockbusters to common programs in computers. Therefore, based on the general understanding and analysis of digital art design, I have formed my personal analysis and opinions on its creation. The hidden formula (5) is as follows:

(5) $$\begin{array}{c} C=M^{2}\text{mod }n. \end{array}$$

The article "Interpretation of Online Artworks of Digital Art Design in the New Media Environment" was published in 2022. Journal: J Environ Public Health.

## 4. Results and Analysis

### 4.1. Promote the Thinking of Aesthetic Works in the New Media Environment

Facing the tradition of realism, some people will question that the expression of digital virtual aesthetics in the form of digital technology and new media art seems to be farther and farther away from real life itself. However, the image world presented by digital aesthetics is imagined and created by people as subjects in the final analysis. The stimulation of people's imagination by virtual aesthetics can not only open up more possibility space for human beings but also meet people's spiritual needs, the spiritual needs of “virtual consumption,” “imagination consumption,” or “symbolic capital consumption.” As another dimension of image documentary online art, there is no doubt about the rationality of the spiritual demand of this kind of consumption. In the “postepidemic era,” this kind of consumption will grow rapidly.  Figure 17 is a graph of the rise of digital technology. Of course, although the rise of digital virtual technology and theorists' theories on “material reality restoration theory,” “realism” film view, and “asymptote” of reality have encountered challenges, films, documentaries, and art films with realism and realistic themes that can be explained by such theories will also exist for a long time. The development of art cannot be judged simply by the theory of evolution in the biological sense [26]. The relationship between art and technology, humanities and science, and technology is undoubtedly very complex, which cannot be covered by either evolution theory or value judgment. There is no doubt that the development of new media art with Internet media as the medium and digital technology as the driving force enriches and expands the territory of art, rather than reducing or splitting art. From a certain point of view, the vitality of art is contained in its huge inclusiveness and expanding territory. As shown in Figure 18, the trend chart of solving problems under new media digital technology is shown. Therefore, it is required that the construction of art theory should not only keep pace with the times, face, pay attention to, and try to solve all kinds of new problems but also be inclusive, commit to the “expansion” of art theory system, and then accommodate all kinds of contradictions and conflicts in an open art theory system and framework. Such an art theory system is open and vigorous. The tree of art is evergreen, and the vitality of art theory is with art.

The article "Interpretation of Online Artworks of Digital Art Design in the New Media Environment" was published in 2022. Journal: J Environ Public Health.

### 4.2. Promote the Interpretation of Aesthetic Works in the New Media Environment

After more than 100 years of development, Chinese aesthetic thought and art theory have made great progress, cultivated many people who are good in both China and the west, and appeared as classic aesthetic works in the field of aesthetics and art history. However, looking at the development history of aesthetic art and the publishing history of aesthetic art theory works, we also face many problems that need to be solved urgently. The above are what most mainstream navigation devices lack at present, which is the significance of designing this system. Nowadays, what the audience needs most for the drama experience is to give the audience the opportunity or space to experience. Otherwise, the audience's drama interpretation is impossible, and the experiential online art is even more on paper. The essence of “unfinished space” is to breed opportunities for the audience's drama experience, provide space for the audience's online interpretation, and enable the audience to actively experience drama in this kind of drama space. And under the organic brewing of drama creators, attract and summon the audience to enter the unfinished space form of drama experience, and this unfinished space state will be open, continuous, and even never complete (and cannot be completed). Its purpose is to constantly breed an updated online art space and attract and summon more viewers' new experience, creation, and perception.  Figure 19 shows the growth of artworks under new media digital technology and the comparison with traditional art interpretation so as to trigger and develop new propositions, new exploration, and new atmosphere of new media drama. This open characteristic of “unfinished space” is undoubtedly a high-quality soil for online interpretation of art.  Figure 20 is a comparison of interpretation of traditional artworks and interpretation of online artworks.

## 5. Conclusion

Chinese aesthetic thought and art theory began at the end of the 19th century and the beginning of the 20th century. The centennial development history of Chinese aesthetic thought and art theory is not only a process of self-construction by absorbing western aesthetic and art resources but also a period of coexistence of various aesthetic thoughts and schools. In this century of development, works on aesthetic art theory have been published continuously, which not only represents the research results and development status of China's aesthetic thought and art theory in different stages but also has important enlightenment significance for the development of later aesthetic thought and art theory. The transformation of digital technology and Internet media is another “holographic” extension of the human body, which has an extremely strong impact on new media art and comprehensively updated our life, art, and aesthetic concepts. This is not only a revolution of media but also a change of art. At the same time, it is also accompanied by the “expansion” of art theory. What this change ultimately needs to complete is the revolution of media culture that affects the development process of human civilization. Media culture “constructs our daily life and ideology and shapes our ideas about ourselves and others; it restricts our values, emotions, and understanding of the world; it constantly makes use of high and new technology and appeals to market principles and universal nonpersonalized audiences. In a word, media culture condenses communication and culture into a dynamic process and coerces everyone.

The article "Interpretation of Online Artworks of Digital Art Design in the New Media Environment" was published in 2022. Journal: J Environ Public Health.

## Figures and Tables

**Figure 1:** Analysis of digital self-media in the field.

**Figure 2:** New media operation flowchart.

**Figure 3:** Composition of new media digital team.

**Figure 4:** Overall market scale of new media server.

**Figure 5:** Professional and understanding of online art interpretation.

**Figure 6:** Crisis management module diagram.

**Figure 7:** Online art appreciation.

**Figure 8:** Problems of modern digital media art design.

**Figure 9:** Schematic diagram of test and evaluation module.

**Figure 10:** Schematic diagram of user communication module.

**Figure 11:** Function module diagram of background management module.

**Figure 12:** Balance principle of online artworks.

**Figure 13:** Recent online art creation.

**Figure 14:** Artistic image of online artworks.

**Figure 15:** Audience satisfaction survey of new media art interpretation.

**Figure 16:** Comparison of reading volume between dramatic artworks and previous works.

**Figure 17:** Rise curve of digital reading technology.

**Figure 18:** Trend chart of problem-solving under new media digital technology.

**Figure 19:** Growth of artworks under new media digital technology.

**Figure 20:** Comparison between interpretation of traditional artworks and online artworks.

## Data Availability

The labeled dataset used to support the findings of this study is available from the author upon request.
